The article "Hedgehog pathway permissive conditions allow generation of immortal cell lines from granule cells derived from cancerous and non-cancerous cerebellum" was retracted in 2020. Reasons: no approval from the institution; copyright claims.

# Hedgehog pathway permissive conditions allow generation of immortal cell lines from granule cells derived from cancerous and non-cancerous cerebellum

**DOI:** 10.1098/rsob.180145

**Published:** 2019-01-09

**Authors:** Constantin Heil

**Affiliations:** Department of Molecular Medicine, University of Rome, ‘La Sapienza’, Rome, Italy

**Keywords:** sonic hedgehog, medulloblastoma, neurosphere, biological assay, granule cells, cell culture

## Abstract

Cerebellar granule cell progenitors (GCPs) undergo proliferation in the post-natal cerebellum that is dependent on sonic hedgehog (SHH) signalling. Deregulated SHH signalling leads to type 2 medulloblastoma (MB). In this work, a novel cell culture protocol is described, which is suitable for the establishment and long-term maintenance of GCP-derived cells. This method is first applied to SHH pathway active MB cells from *Atoh1*-cre;*Ptch1*^FL/FL^ tumours, which leads to the generation of neurosphere-like cell lines expressing GCP markers and an active SHH signalling pathway. These cells also show high sensitivity to the Smoothened inhibitor vismodegib, therefore recapitulating the SHH pathway requirement for survival shown by type 2 MB. Analysis of culture supplements reveals that bFGF and fetal bovine serum act as inhibitors of the SHH pathway and therefore preclude generation of cell lines that are relevant to the study of the SHH pathway. Consequently, these insights are transferred from the context of MB to non-transformed, post-natal day 7 cerebellum-derived cellular explants. In contrast to other, previously used methods, these GCP cultures proliferate indefinitely and depend on SHH pathway activation, either by means of the small molecule SAG or through genetic ablation of *Ptch1*. This culture method therefore leads to the generation of immortal neurosphere-like cell lines, that are named murine SAG-dependent spheres (mSS). Despite long-term culture, mSS cells remain dependent on continuous stimulation of the SHH pathway. Further, mSS cells maintain their lineage after extensive periods *in vitro,* as demonstrated by their differentiation towards the neural lineage. Herein a simple method for the generation of immortal cell lines from murine cerebella is defined. These lines can be maintained indefinitely through hedgehog pathway activation and maintain the GCP lineage.

## 1. Introduction

Cell culture technologies are used in biomedical research as well as developmental biology to conduct experimentation on controllable and scaleable systems. Among the different biomedical fields, cancer research makes extensive use of cell cultures. The first human cells to be stably cultured were cancer cells and to this day most cell lines in use derive from human cancer [1]. Further, cancer cell lines are used extensively in pre-clinical research and are the basis for other technologies such as high-throughput screening or other biological assays [2,3].

The article "Hedgehog pathway permissive conditions allow generation of immortal cell lines from granule cells derived from cancerous and non-cancerous cerebellum" was retracted in 2020. Reasons: no approval from the institution; copyright claims.

Cells used *in vitro* can be distinguished based on their persistence in culture. Primary cells can generally be passaged a limited number of times before undergoing crisis [4], while transformed cells are characterized by autonomous unlimited proliferation. Immortalized, yet non-transformed cells can be considered intermediate between these two aforementioned cell types in that they possess the capability for unlimited expansion while maintaining key properties of the original tissue, such as lineage and differentiation capabilities [5]. Commonly used immortal cell lines used in developmental biology are C17.2 cells [6] and C2C12 cells [7]. Another commonly used method for culture of neural progenitors is the neurosphere method [8], wherein cells are cultured in defined serum-free medium and proliferate as floating spheres. Neurospheres can be cultured indefinitely and were initially characterized as stem cells; however, more recent findings call into question whether neurospheres are bona fide stem cells or so-called transit amplifying cells [9].

In addition to the origin of cultured cells, the relevance of *in vitro* systems towards modelling a biological process depends on how accurately cell culture conditions recreate an environment in which those cells maintain the properties of interest. In the case of cancer cell lines, these properties tend to be related to key behaviours of the tumour, i.e. extensive proliferation, migration or refractivity to differentiation [5], but also activity and dependence on key oncogenic pathways. In any case, cell culture systems are artificial models of biological processes, with the culture medium and the cells therein being two interacting components. Importantly, the culture medium plays the role of an environment that selects for a ‘fit’ subset of cells originally plated. It therefore follows that the composition of culture medium plays an important role towards conditioning the properties of the cells cultured therein.

During the development of the mammalian cerebellum, a post-natal expansion of cerebellar granule cell progenitors (GCPs) generates the population of mature granule neurons of the cerebellar cortex. These cells proliferate in the external granule layer (EGL) of the cerebellar anlage and continuously differentiate and migrate radially to the internal granule layer (IGL) of the cerebellar cortex [10]. A key mitogen for GCPs in the EGL is sonic hedgehog (SHH) [11,12], which is secreted by underlying Purkinje neurons. SHH is necessary and sufficient for the expansion of the GCP compartment. Further, defects in SHH signalling lead to aberrant proliferation that culminates in the paediatric cancer type 2 medulloblastoma (MB) [13–15]. Cells of type 2 MB show a characteristic gene expression pattern that overlaps with GCPs in terms of key signalling pathways and proliferation associated genes [15]. For example, GCPS as well as type 2 MB cells express the lineage-specific ATOH1 and components of the activated SHH pathway such as GLI1, PTCH1 and NMYC.

The article "Hedgehog pathway permissive conditions allow generation of immortal cell lines from granule cells derived from cancerous and non-cancerous cerebellum" was retracted in 2020. Reasons: no approval from the institution; copyright claims.

Various cell culture conditions have been applied to GCPs or type 2 MB cells. GCPs are generally cultured as adhesive cell cultures. These cultures recapitulate the SHH signalling requirement for GCP proliferation [12,16]. Importantly, GCPs cultured in this way will eventually cease proliferation even in the presence of an SHH pathway agonist [12], therefore recapitulating the transient proliferation that these cells undergo *in vivo*. Type 2 MB cells have been cultured in various ways. While human MB cells, which are also used to study the SHH pathway [17], are generally cultured in DMEM supplemented with FBS, it has been demonstrated that murine cells cultured in this way lose the activity of the SHH pathway [18]. Another method that is applied to murine type 2 MB model-derived cells is their culture under the previously mentioned neurosphere conditions that are presumed to enrich for stem-like cells [19]. In short, there are various challenges involved in modelling the different facets of the GCP lineage *in vitro*. Primary GCP cultures recapitulate key properties of the lineage, yet their transientness limits the amount of sample obtainable while requiring a constant supply of animals. This can be limiting for ethical or logistic reasons. While tumour-derived cells can be cultured persistently, the transformed nature of the original sample may make it difficult to study properties relevant to physiological processes such as differentiation. Further, culture methods themselves may modify the status of the SHH signalling pathway.

In this work, culture methods for cells of the GCP lineage are explored. These cells are either derived from normally developing cerebella or models of type 2 MB. By identifying commonly used factors that inhibit the expression of the SHH pathway *in vitro* and subtracting these factors from the medium, a protocol for the long-term culture of either transformed or non-transformed GCP cells is obtained.

## 2. Results

### 2.1. Generation of relevant murine tumour spheres from a conditional knockout disease model

It was recently reported that murine primary MB explants from the *Ptch1*^+/−^ model could be cultured as tumour spheres that maintain the activity of the SHH pathway [20]. This approach is applied to another model of murine SHH type MB, the *Atoh1*-cre;*Ptch1*^FL/FL^ mouse. As reported previously, cells proliferated in the form of floating spheres.

The article "Hedgehog pathway permissive conditions allow generation of immortal cell lines from granule cells derived from cancerous and non-cancerous cerebellum" was retracted in 2020. Reasons: no approval from the institution; copyright claims.

These cells, herein named SHH medulloblastoma tumour spheres (MBSHH-TS), express relevant lineage-specific and SHH pathway-associated genes and consequently cluster together with their respective primary tumour tissues of origin (figure 1*a*), as demonstrated by hierarchical clustering. Conversely, MBSHH-TS cell lines are readily distinguishable from the distinct type 4 MB model GTML. MBSHH-TS cells further demonstrated nanomolar sensitivity to 24 h of treatment with the Smoothened inhibitor vismodegib, as shown by XTT assay (figure 1*b*). To confirm that vismodegib sensitivity is specifically caused by its effect on the SHH pathway, the expression of NMYC and GLI1 proteins is assayed by western blot, both of which decreased in a dose-dependent manner (figure 1*c*). Apoptosis was confirmed by the detection of cleaved PARP1. Expression of *Gli1*, *Ptch1*, *Ptch2* and *Hhip* genes was also assayed by QPCR. All of these genes responded negatively to vismodegib treatment (figure 1*d*). MBSHH-TS cells therefore express an active SHH signalling pathway and are sensitive to treatment with a Smoothened inhibitor, thus recapitulate key disease hallmarks.

**Figure 1.** Properties of medulloblastoma cell lines from *Atoh1*-cre;*Ptch1*^FL/FL^ murine tumours. (*a*) Heatmap summarizing QPCR data comparing MBSHH-TS cell lines with their respective original tumours and with GTML murine medulloblastomas. (*b*) XTT assay measuring vitality of MBSHH-TS cells as function of vismodegib dosage. *X*-axis is base 10 logarithm of mM. *n* = 3. (*c*) Western blot measuring levels of GLI1, cPARP1 and NMYC in response to different vismodegib dosages. Presented blot is representative of *n* = 3 replications. (*d*) QPCR data depicting SHH pathway gene expression levels after vismodegib treatment. *n* = 3. (*e*) Comparison of GLI1 and ZIC1 protein levels between MB-EF and MBSHH-TS cells originating from same initial tumour. (*f*) GLI1 and NMYC protein levels in MBSHH-TS cells after exposure to either bFGF of fetal bovine serum (FBS). Presented blot is representative of *n* = 3 replications.

To analyse the emergence of these relevant cell lines, explants deriving from the same *Atoh1*-cre;*Ptch1*^FL/FL^ tumour were cultured in neurosphere medium with or without supplementation of EGF and bFGF, termed MB-EF cells. In both cases, cell lines emerge; however, MB-EF cells do not express detectable levels of either GLI1 or ZIC1 protein after one month *in vitro* (figure 1*e*). The finding that growth factors may not support SHH signalling reflects literature that describes that bFGF treatment inhibits the signalling pathway [21]. Consistent with these observations, treatment of established MBSHH-TS cells with either bFGF or serum for 24 h led to the diminishment of GLI1 protein expression and the SHH pathway downstream effector NMYC (figure 1*f*).

The article "Hedgehog pathway permissive conditions allow generation of immortal cell lines from granule cells derived from cancerous and non-cancerous cerebellum" was retracted in 2020. Reasons: no approval from the institution; copyright claims.

### 2.2. The post-natal cerebellum supports the generation of novel neurosphere cultures that express an activated SHH pathway

In the context of the forebrain, the discovery that cells could be cultured as neurospheres eventually led to another interesting discovery. That is, brain tumours, such as glioblastoma multiforme (GBM), could also give rise to neurosphere cultures [22]. This suggests that cells from the same lineage can be cultured under the same cell culture conditions, regardless of their status of being transformed or not.

To explore the possibility that this commonality between diseased and physiological states could be extended from the context of SHH type MB to non-transformed GCP cells, it can be conjectured that cells originating from non-tumourous post-natal murine cerebellar explants should be cultured under conditions that support SHH pathway activation. To investigate this conjecture, cell pools originating from dissociated post-natal day 7 (p7) murine cerebella were exposed to serum-free neurosphere culture conditions, supplemented with the growth factors bFGF and EGF (EF conditions) and/or SAG, a small molecule agonist of the SHH signalling pathway [23].

After 7 days in culture, primary cerebellar explants treated with EF conditions lost expression of the SHH pathway mediator GLI1 while cells exposed to SAG maintained GLI1 expression (figure 2*a*). Further, GLI1 expression is also undetectable in cells exposed to EF together with SAG, thus confirming previous observations that growth factor signalling can actively inhibit SHH signalling. In addition to measurement of GLI1 and NMYC protein levels, clonogenicity was measured in order to confirm the functional effects of the different treatments. All treatments led to comparable clonogenicity, while control (DMSO)-treated cells did not give rise to clones (figure 2*b*). In order to assess the magnitude of SHH signalling in SAG-cultured explants, their levels of expression of key SHH pathway members were compared with those of murine cerebellum at phases of GCP proliferation (p5) and quiescence (p21). SAG-exposed explants expressed significantly higher levels of the SHH pathway mediators *Gli1*, *Gli2* or *Nmyc* (figure 2*c*).

The article "Hedgehog pathway permissive conditions allow generation of immortal cell lines from granule cells derived from cancerous and non-cancerous cerebellum" was retracted in 2020. Reasons: no approval from the institution; copyright claims.

**Figure 2.** Generation of novel SHH pathway active neurospheres from murine cerebellum. (*a*) Western blot of different primary cultures after 7 days in culture. Presented blot is representative of *n* = 3 replications. (*b*) Clonogenicity of explants as in (*a*) and control (DMSO)-treated explants. (*c*) QPCR detection of *Gli1, Gli2* and *Nmyc* in p5 cerebella, p21 cerebella and cerebellar explant at seven days *in vitro* with SAG. *n* = 3. (*d*) Clonogenicity of SAG cultured cells exposed to different concentrations of SAG. (*e*) Boxplots presenting sphere diameters of cells treated as in (*d*). (*f*) QPCR of different established cell types and YAC1 mouse lymphoblastoid cells for detection of *Nestin*, *Sox2*, *Pou5f1* and *Pou3f2* levels. *n* = 3. (*g*) Serial clonogenic assay carried out each week, over a period of 10 weeks, from SAG cultured explants. Micrograph represents established mSS cells. (*h*) Boxplots present sphere diameters from early passage cultures (two weeks *in vitro*) of established mSS lines (10 weeks *in vitro*).

After having established SHH pathway expressing neurospheres, primary cerebellar explants were challenged with a lower dose of SAG to investigate sensitivity to SAG levels. Reducing the dose to 0.2 µM SAG led to significantly decreased sphere formation from primary cerebellar cells (figure 2*d*). SAG treatment also causes a similar dose dependent effect on sphere size, which is a measurement of the cell division rate within the sphere (figure 2*e*).

It has been previously reported that SAG can act as an inhibitor of Smoothened at concentrations around 1.0 µM [23]. In order to address this possibility for a relevant range of concentrations of SAG, doses of SAG up to 1.0 µM were applied to determine if they could inhibit the basal proliferation of primary *Atoh1*-cre; *Ptch1*^FL/FL^ cells (electronic supplementary material, figure S6). No inhibition of constitutive proliferation was observed at 1.0 µM, nor was there any inhibition of any hypothetical growth increment that may occur at lower doses of SAG.

To assess whether these novel SAG-exposed neurospheres recapitulate the expression of neural progenitor-associated genes, as observed for other neurosphere types [24], *Nestin*, as well as the stem-cell factors *Sox2* and its binding partners *Pou5f1* (also referred to as *Oct4*) and *Pou3f2* (also referred to as *Brn2*) were assayed in comparison with the murine lymphoblastoid line YAC1 and EF established neurospheres from the same explant at two weeks *in vitro*. SAG-exposed cells expressed all the aforementioned markers, even if *Sox2* was expressed at lower levels with respect to mEF cells (figure 2*f*).

The article "Hedgehog pathway permissive conditions allow generation of immortal cell lines from granule cells derived from cancerous and non-cancerous cerebellum" was retracted in 2020. Reasons: no approval from the institution; copyright claims.

In addition to the expression of stem-cell-associated genes, neurospheres are known for their extensive proliferative capability, while GCP cultures have normally been described as being of transient nature, consistent with their developmental origin. To investigate this property in SAG-cultured cells, their long-term proliferative properties were challenged by measuring clonogenicity for a period of 10 weeks, corresponding to 20 passages. This experiment reveals that SAG supports continuous clonogenicity of these cells throughout the duration of the experiment (figure 2*g*). Further, clonogenic potential as well as sphere diameter (figure 2*h*) remain stable throughout the course of 10 weeks. In conclusion, two important parameters of cell proliferation remain unaltered by long-term culture.

The fact that SAG-stimulated cerebellar explants give rise to neurosphere cultures with extensive proliferative capability allows the establishment of permanent cell lines through this method. From this point, such established lines that have been in culture for at least 10 weeks will be referred to as murine SAG-dependent spheres (mSS), while their associated neurosphere lines, cultured in EGF and bFGF will be referred to as mEF.

### 2.3. Hedgehog pathway active, cerebellum-derived neurospheres belong to the GCP lineage

Murine neurospheres have been shown to originate from diverse sites along the neuraxis such as the sub-ventricular zone (SVZ). To investigate the specificity of the establishment of SAG-dependent neurospheres as a function of anatomic location, SVZ and cerebellar explants from p7 brains were exposed to either EF conditions or SAG and sphere formation was assayed in terms of clonogenicity.

While the observation that neurospheres can be obtained from the SVZ and cerebellum in the presence of the two growth factors was replicated [25], SAG could only stimulate the generation of neurospheres from the cerebellum (figure 3*a*). This observation suggests that the *in vivo* origin of these cells could be a cell type unique to the cerebellum at this developmental stage.

**Figure 3.** mSS cells belong to the GCP neurogenic lineage. (*a*) Clonogenic assay carried out using explant cells from different sources (SVZ and cerebellum) and exposed to different treatments (SAG and EGF/bFGF). (*b*) Western blot showing GLI1 and ZIC1 protein levels (i) and QPCR to assay *Atoh1* levels (ii) in EGF/bFGF and SAG exposed cultures throughout the duration of one month in culture. Presented blot is representative of *n* = 3 replications, for QPCR *n* = 3. (*c*) Clonogenic assay carried out with explants from either wild-type (WT) or *Ptch1* conditional knockout cerebella. (*d*) Comparison of gene expression by QPCR between mEF, mSS and mPS cells. Data presented for *Gli1*, *Gli2*, *Nmyc*, *Ptch1*, *Atoh1*, *Zic1*, *Ccnd2* and *Pax6*. *n* = 4. All differences mSS versus mEF are significant. Numbers represent *p*-values for the comparison of mSS versus mPS.

The article "Hedgehog pathway permissive conditions allow generation of immortal cell lines from granule cells derived from cancerous and non-cancerous cerebellum" was retracted in 2020. Reasons: no approval from the institution; copyright claims.

As proliferating GCP cells are an abundant cell type in the post-natal murine cerebellum, cultures were established under EF conditions or alternatively SAG treatment and the expression of ZIC1 protein and *Atoh1* transcript were monitored during the course of the initial culture, as these are both reported as being markers of the GCP lineage. ZIC1 protein levels gradually decrease under EF conditions, being undetectable after 6 days, while in SAG-treated cultures ZIC1 levels stabilize after one month, concomitant with increased levels of GLI1 (figure 3*b*(i)). Concordantly, *Atoh1* transcript levels were gradually enriched in SAG-exposed cells while they gradually decreased under EF conditions (figure 3*b*(ii)). The gradual increase in GCP lineage markers, of which *Atoh1* and *Zic1* are not transcriptionally activated by the SHH pathway [16,17], in SAG-exposed cells suggests the enrichment of GCP cells at the expense of SAG non-responsive cells. This idea is supported by the gradual accumulation of GLI1 protein, reflecting the explant's gradual evolution from a heterogeneous, tissue-derived cell suspension to a more homogeneous cell line under the selective stimulus of mitogenic SAG.

To further confirm that SAG-responsive cells are of the GCP lineage, SAG treatment was substituted with genetic activation of the SHH signalling pathway in the GCP lineage. In *Atoh1*-cre;*Ptch1*^FL/FL^ mice, *cre* recombinase expression is driven in cells of the GCP lineage [26]. Clonogenic assay was carried out on cells originating from p7 cerebella of either *Atoh1*-cre;*Ptch1*^FL/FL^ mice or wild-type litter mates and clonogenicity was observed with SAG treatment, while only conditional knockout (KO) cells gave rise to spheres in the absence of SAG (figure 3*c*), which will be referred to as murine *Ptch1* KO-derived spheres (mPS) after the establishment as a long-term (minimum ten week) cell line. In conclusion, it seems likely that cells of the GCP lineage respond to SAG treatment with SHH signalling pathway activation and proliferation under these conditions. To further establish the identity of the GCP-derived cell lines with respect to mEF neurospheres, expression of key SHH pathway components (*Gli1*, *Gli2*, *Nmyc*, *Ptch1, Ccnd2*) and GCP lineage markers (*Atoh1*, *Zic1, Pax6*) was assayed. Expression of these markers was very low in mEF cells, with respect to mSS or mPS cells. Further, expression levels of the genes were similar between mSS and mPS cells, except in the case of the genes *Gli2* and *Nmyc,* possibly due to differences in the strength of SHH signalling activation between pharmacological and genetic activation of the pathway.

The article "Hedgehog pathway permissive conditions allow generation of immortal cell lines from granule cells derived from cancerous and non-cancerous cerebellum" was retracted in 2020. Reasons: no approval from the institution; copyright claims.

### 2.4. mSS cells continuously require SHH pathway stimulation

To assay the continuous requirement for Smoothened stimulation for SHH pathway activation and proliferation of mSS cells, these cells were treated with either KAAD-cyclopamine or vismodegib, inhibitors of the Smoothened protein, for a duration of 24 h. Consistent with the above observations, inhibitor treatment leads to the downregulation of SHH pathway components in terms of transcript and protein levels (figure 4*a*(i,ii), respectively). This reduction of SHH pathway activation was also concomitant with loss of clonogenicity in the case of both inhibitors (figure 4*b*).

**Figure 4.** Established mSS cell lines maintain dependence on SHH pathway. (*a*) QPCR (i) and western blot (ii) assaying SHH pathway members in mSS cells after Smoothened inhibitor treatment. Presented blot is representative of *n* = 3 replications, for QPCR *n* = 3. (*b*) Clonogenic assay in Smoothened inhibitor treated mSS cells. (*c*) Clonogenic assay on long-term cultured mSS cells upon deprivation from SAG supplementation.

The continuous requirement for pharmacological activation of the SHH could also be demonstrated by removing SAG, as opposed to treating with a Smoothened inhibitor. Towards this end, cells were spinned down and washed in PBS before being dissociated and re-plated for clonogenic assay in either SAG, DMSO or vismodegib. DMSO-treated cells showed a marked decrease in clonogenic potential (figure 4*c*), therefore confirming the requirement for Smoothened activation.

### 2.5. mSS cells maintain neural lineage commitment after long-term culture

It has been reported that the plasticity of neural progenitors can be modified after long periods of time in cell culture [27]. To assay the *in vitro* differentiation capabilities of mSS cells, paired mSS and mEF neurospheres were plated in medium containing serum, a condition reported to promote neurosphere differentiation towards the astrocytic lineage [28]. Both cell types attached to the dish within 24 h and after 5 days in these conditions mSS cells acquired an elongated bipolar neuronal morphology while mEF neurospheres acquired a stellate glial morphology (figure 5*a*).

**Figure 5.** Established mSS lines maintain neurogenic differentiation potential. (*a*) Phase-contrast microscopy photo of mSS and mEF cells at 1 day or 5 days in differentiation conditions. Scale bar corresponds to 100 µm. (*b*) (i) Immunofluorescence for TUBB3 or GFAP in mSS or mEF cells at 5 days in differentiation conditions. Scale bar corresponds to 100 µm. Histograms (ii) express relative numbers of each cell type. (*c*) (i) Western blot comparing beta3-tubulin (TUBB3) or GFAP levels between 5-day differentiated mSS or mEF cells. (ii) QPCR of *Atoh1* and *Gabra2* in differentiated mSS cells. Presented blot is representative of *n* = 4 replications. For QPCR, *n* = 3.

The article "Hedgehog pathway permissive conditions allow generation of immortal cell lines from granule cells derived from cancerous and non-cancerous cerebellum" was retracted in 2020. Reasons: no approval from the institution; copyright claims.

In addition, mEF and mSS cell cultures were analysed by immunofluorescence (IF) for TUBB3 (beta3-tubulin) and GFAP, markers of the neural and glial lineages, respectively. mEF cells gave rise to a homogeneous population of GFAP positive cells while mSS cells gave rise to an overwhelming majority of TUBB3 staining cells (figure 5*b*). Subsequently, TUBB3 and GFAP levels were also measured by western blot. In agreement with the above mentioned morphological changes and IF data, mSS cells upregulated expression of TUBB3; on the other hand, mEF neurospheres expressed high levels of GFAP under these conditions (figure 5*c*, top).

After having established neuronal lineage commitment for mSS cells, expression of *Gabra2* and *Atoh1* was quantified in differentiated cells. In agreement with the GCP identity of mSS cells, *Atoh1* transcript levels decreased, while *Gabra2* levels accumulated upon differentiation (figure 5*c*(ii)).

## 3. Discussion

This work establishes a method for the culture of murine cells that belong to the GCP lineage. Notably, this method can be applied to different GCP originating cells, in the sense that the same method establishes cultures from transformed and non-transformed cells of the GCP lineage.

Initially, a previously published method [20] is applied to a different model of murine MB. The validity of the approach is confirmed also in the case of the *Atoh1*-cre;*Ptch1*^FL/FL^ genotype and the analysis is extended towards understanding how commonly used cell culture supplements influence the SHH pathway. It is demonstrated that both bFGF and fetal bovine serum (FBS) act as inhibitors of the SHH pathway. Based on these observations, commonly used supplements to cell culture are confirmed to act as inhibitors of the SHH pathway and should be avoided in this context.

The inhibitory effects of aforementioned supplements on SHH signalling suggest that those cells that do emerge under these conditions do not require the mitogenic effect of the pathway and therefore their relevance for the study of the SHH pathway is questionable. While this problem was previously treated in Sasai *et al.* [18], in which the authors observe that culturing cells obtained from murine MB models in DMEM supplemented with FBS led to establishment of stable lines despite inhibition of the SHH pathway, this research broadens the concept that a cell line may not necessarily represent key properties of its originating tissue when culture conditions are not favourable.

The article "Hedgehog pathway permissive conditions allow generation of immortal cell lines from granule cells derived from cancerous and non-cancerous cerebellum" was retracted in 2020. Reasons: no approval from the institution; copyright claims.

Other commonly used cell models of SHH signalling are murine 3T3 cells and human DAOY MB cells. In both of these cell types, SHH activity is coerced from these cells by placing them in conditions of low serum at high confluency [17,23]. These conditions render the study of cancer relevant readouts, such as proliferation, difficult and they cast doubt on the specificity of the relationship between the cell's origin and its SHH signalling status. The effect of SHH pathway inducibility and cell confluence may be cell-type aspecific and mediated by the YAP pathway [29].

After establishing conditions that allow for the generation of SHH pathway active neurospheres from murine cerebellum, it is observed that these cells possess the capability for unlimited proliferation. Therefore, while previous culture methods of GCP cells led to cultures that were transient even when the SHH pathway was activated [12,13], this work describes a method for establishing stable GCP cell lines, herein named mSS. An important property of mSS cells is their ability to undergo long-term proliferation without immortalization through exogenous oncogenes, such as is the case for C17.2 cells [6], that derive from murine cerebellum and carry the *v-myc* oncogene. This is significant because immortalization through oncogenes has been reported to modify the lineage of GCPs [30]. Unlimited growth as neurospheres of physiologically transit amplifying cells has previously also been observed within the lineage of the SVZ [9].

Interestingly, when considered in comparison with conventionally established neurosphere cultures, mSS cells express lower levels of ‘stemness' associated genes *Sox2* and *Nestin,* which are, conversely, undetectable in tumour cells. This is consistent with the identity of mSS cells belonging to the GCP lineage, as GCPs are more committed progenitors with respect to multi-potent stem cells [10].

mSS cells can be considered immortal cell lines that continuously recapitulate the relevant properties of their tissue of origin. These cell lines remain dependent on exogenous growth stimulus in the form of SAG and maintain the ability for differentiation towards only the neural lineage, thus being by definition immortalized and not transformed. Additionally, the growth properties of mSS cells, measured in terms of clonogenicity and sphere size, do not vary over time. In this sense, mSS cells are similar to the aforementioned C17.2 cells or C2C12 myoblastic cells [7] for the field of myogenesis, extensively expandable and differentiable on demand.

The article "Hedgehog pathway permissive conditions allow generation of immortal cell lines from granule cells derived from cancerous and non-cancerous cerebellum" was retracted in 2020. Reasons: no approval from the institution; copyright claims.

## 4. Protocol

### 4.1. Establishment

(1) Sacrifice p7 murine pups by decapitation. Take into consideration that each cerebellum at this stage will give around 3 × 10^6^ platable cells. Final density will be 62 500 cells ml^−1^, i.e. 750 000 cells for a 12 ml culture in a T75 flask.
(2) Use one pair of fine forceps to cut away the skin from the posterior neck upwards, thus exposing the occipital cranium. Use another pair of forceps to repeat the same cut, but applied to the cranium to expose the cerebellum. It is advised to use different forceps for each cut so as not to carry over skin contaminants to the neural tissue.
(3) Isolate the complete cerebellum by pinching it off with curved tweezers and place in 5 ml post-surgery medium (see below).
(4) From now on work under cell culture hood.
(5) Smash the cerebellum with a 5 ml pipette, then pipette up and down repeatedly until the suspension is liquid and homogeneous. Repeat pipetting up and down with a Pasteur pipette, again until the suspension is homogeneous.
(6) Add DNase I to a final concentration of 0.04%, leave at room temperature for 20 min. Counteract sedimentation of cells by inverting tube every 5 min.
(7) Pellet cells at 1000 rpm for 5 min and resuspend 62 500 cells ml^−1^ in cell medium (see below).
(8) Pass cells by spinning down at 1000 rpm and resuspending in medium. It is advised to split by a factor of two every two or three days.

### 4.2. Differentiation

(1) Spin down neurospheres and resuspend in differentiation medium. Pipette up and down to dissociate spheres. Do not dissociate completely or use enzymatic dissociation methods as this will greatly diminish viability.
(2) Plate cells on polylysinated cell culture dishes.

### 4.3. Media

Cell medium

DMEM/F12

0.6% glucose

25 µg ml^−1^ insulin

60 µg ml^−1^ *N*-acetyl-l-cysteine

2 µg ml^−1^ heparin

1 × penicillin/streptomycin

1 × B27 supplement without vitamin A

1 µM SAG

Post-surgery medium

Hanks' balanced salt solution (HBSS)

0.5% glucose

1 × penicillin/streptomycin

Differentiation medium

Neurobasal

1 × glutamine

1 × penicillin/streptomycin

0.5% FBS

B27 supplement (with vitamin A)

## 5. Conclusion

Various *in vitro* systems are used to study the SHH pathway in the context of cerebellar GCP biology. These are either cell lines that are used to study the SHH pathway in a context-independent manner, such as NIH3T3 cells, or primary GCP cultures, which are a contextually more relevant model. NIH3T3 cells do not belong to the neural lineage and require pre-treatment before being reactive to SHH pathway activation while primary GCP cultures are transient and therefore can constitute a bottleneck for generation of sample material. A more persistent method of cell culture for GCP lineage would also be important for ethical reasons, as the number of sacrificed animals could be greatly diminished.

The article "Hedgehog pathway permissive conditions allow generation of immortal cell lines from granule cells derived from cancerous and non-cancerous cerebellum" was retracted in 2020. Reasons: no approval from the institution; copyright claims.

In this paper, a generalized protocol for the culture of cells of the GCP lineage is proposed. It is demonstrated that commonly used cell culture supplements inhibit the SHH pathway, therefore precluding the establishment of relevant GCP lines. This protocol, on the other hand, is permissive to continuous activity of the SHH pathway, which is mitogenic for cells of this lineage. It therefore follows that this protocol establishes long-term cultures from normal p7 cerebella or murine models of type 2 MB. The MB-derived cells are named MBSHH-TS and it is reported that these cells recapitulate disease-relevant properties, such as expression of relevant markers and sensitivity to Smoothened inhibitors. Further, the cell culture paradigm is extended to non-cancerous GCP cells. These cells are named mSS, and it is demonstrated that they are valid models for cerebellar neurogenesis as they proliferate indefinitely under the condition of genetically or pharmacologically activated Smoothened. Further, mSS cells differentiate *in vitro* into granule neurons. The establishment of these cell lines is reproducible and relatively simple, and therefore constitutes a useful methodology for the study of the SHH pathway or cerebellar neurogenesis.

## 6. Material and methods

### 6.1. Establishment of cultures from murine central nervous system

Post-natal day 7 (p7) mice were sacrificed by decapitation and tissues were collected in HBSS supplemented with 0.5% (w/v) glucose and penicillin/streptomycin, grossly triturated with a serological pipette and treated with DNAse I to a final concentration of 0.04% (w/v) for 20 min. Finally, cell aggregates were mechanically dissociated using pipettes of decreasing bore size to obtain a single-cell suspension. After centrifugation, single cells were cultured as neurospheres in selective medium: DMEM/F12 supplemented with 0.6% (w/v) glucose, 25 µg ml^−1^ insulin, 60 µg ml^−1^ *N*-acetyl-l-cysteine, 2 µg ml^−1^ heparin, 20 ng ml^−1^ EGF, 20 ng ml^−1^ bFGF (Peprotech, Rocky Hill, NJ) or 1 µM SAG (Adipogene), 1× penicillin/streptomycin and B27 supplement without vitamin A. SAG dosage was 1 µM unless otherwise specified. For a more detailed description of the method, see the Protocol section.

For differentiation, cells were mechanically dissociated and plated on polylysinated cell culture dishes in the following medium: Neurobasal (Invitrogen) supplemented with glutamine, penicillin/streptomycin, 0.5% (v/v) FBS and B27 supplement.

The article "Hedgehog pathway permissive conditions allow generation of immortal cell lines from granule cells derived from cancerous and non-cancerous cerebellum" was retracted in 2020. Reasons: no approval from the institution; copyright claims.

Cells can be cryopreserved at −80°C in BAMBANKER serum-free cryopreservation medium (Wako Pure Chemical Industries, no. 306-95921)

XTT assays were carried out using Roche Cell Proliferation Kit II (no. 11465015001)

### 6.2. Clonogenic assay

Cells were pelleted and dissociated by incubation with Accutase (Sigma Aldrich) concomitant with continuous pipetting to obtain a single-cell suspension. Cells were counted with a haemocytometer and were diluted to obtain a suspension of 0.267 cells µl^−1^. The cell suspension was distributed on a 96-well plate, pipetting 75 µl into each well.

Respective treatments were prepared with double the final concentration and 75 µl was added to each well for a final volume of 150 µl at a concentration of 0.134 cells µl^−1^, for a total of 20 cells per well. After 3 days, the medium was replenished and an additional 3 days later the number of spheres per well was recorded. Exhibited data represent averages of two independent experiments, each having 24 wells per treatment point.

### 6.3. RNA preparation and quantitative reverse transcription-PCR

Total RNA extraction was carried out with TRIzol reagent (Invitrogen). For quantitative reverse transcription-PCR (QPCR), total RNA (1 µg) was reverse transcribed using the Gene Amp kit (Applied Biosystems) and subjected to PCR amplification using SYBR Green PCR Master Mix (Applied Biosystems) or TaqMan PCR Master Mix (Applied Biosystems). Samples underwent 40 amplification cycles (95°C for 10 s; 60°C for 1 min) in an ABI Prism 7900 machine (Applied Biosystems). TaqMan probes (Applied Biosystems) were used to detect HPRT, GLI1, PTCH1, GABRA2 and MYCN. For SYBR green QPCR the following primers were used:

Nestin FW GCAGGCCACTGAAAAGTTCC

Nestin RV CACCTTCCAGGATCTGAGCG

SOX2 FW CAGGAGTTGTCAAGGCAGAGA

SOX2 RV CTTAAGCCTCGGGCTCCAAA

POU3F2 FW CCTTTAACCAGAGCGCCCA

POU3F2 RV AGGCTGTAGTGGTTAGACGC

POU5F1 FW GGCTTCAGACTTCGCCTTCT

POU5F1 RV TGGAAGCTTAGCCAGGTTCG

ATOH1 FW CCCGTCAAAGTACGGGAACA

ATOH1 RV CTCGTCCACTACAACCCCAC

The heat maps in figure 1 and electronic supplementary material, figure S6*a* were made using the R package *pheatmap.*

Please note that *Atoh1*-cre;*Ptch1*^FL/FL^ mice are as reported in Ellis *et al.* [26]. In these mice, the *Ptch1* ORF is disrupted; however, an SHH responsive transcript is still produced from the modified locus [26].

### 6.4. Protein extraction and western blot

Total protein extracts were obtained in RIPA buffer (50 mmol l^−1^ Tris (pH 8.0), 150 mmol l^−1^ NaCl, 0.5% (w/v) sodium deoxycolate, 0.1% (w/v) SDS, 1% (v/v) NP40, 0.001 mol l^−1^ EDTA and a mix of protease inhibitors). Protein extracts were separated by SDS-PAGE and blotted onto nitrocellulose membranes (Perkin Elmer). Membranes were blocked with 5% (w/v) nonfat dried milk and incubated with primary antibodies (Abs) at the appropriate dilutions. Abs were as follows: goat anti-β-actin, rabbit anti CCND1 and mouse anti-MYCN (Santa Cruz Biotechnology), mouse anti-Gli1, no. 2643 (Cell Signaling Technology Inc). Immunoreactive bands were visualized by enhanced chemoluminescence (Perkin Elmer).

The article "Hedgehog pathway permissive conditions allow generation of immortal cell lines from granule cells derived from cancerous and non-cancerous cerebellum" was retracted in 2020. Reasons: no approval from the institution; copyright claims.

Densitometric analysis was carried out using ImageJ. Actin normalized optical density results are reported as numbers under the relevant bands and summarized as bar plots in electronic supplementary material, figure S8.

### 6.5. Immunofluorescence

Cells were fixed in 4% (v/v) paraformaldehyde and washed with PBS. Samples were permeabilized in 0.1% (v/v) Triton-X 100 in PBS for 15 min at room temperature, washed in PBS and blocked in 5% (w/v) BSA for 30 min at room temperature. Primary antibodies were diluted in 1% (w/v) BSA, incubated overnight at +4°C and were the following:

mouse anti-GFAP monoclonal antibody MAB360 (Millipore);

mouse anti-neuronal class IIIb-tubulin (TUJ1) monoclonal antibody MMS-435P (Covance).

Samples were washed in PBS and incubated in Alexa Fluor 555 goat anti-mouse (Life Technologies) together with Hoechst nuclear dye for 20 min at room temperature. After further washes in PBS, slides were mounted in PBS/glycerol and analysed under a fluorescence microscope. Images were analysed and scored using ImageJ.

### 6.6. Statistical methods

Unless otherwise indicated, significance was tested using unpaired, two tailed *t*-test without the assumption of equal variance. *p*-Values are reported as *p < 0.05, **p < 0.005, ***p < 0.005, ****p < 0.0005, unless otherwise specified.

Reported values for ‘*n*’ indicate the number of samples per category. ‘*n*’ refers to biological replicates unless otherwise specified.

## Supplementary Material

Supplementary figures

## Data accessibility

Raw data are available in the electronic supplementary material file.
